The article "Correlation Analysis of Adverse Reactions of Antiosteoporosis Drugs by Different Mechanisms with Bone Turnover and Vitamin D" was retracted in 2023. Reasons: unreliable results or conclusions; concerns about the peer review; concerns about the citations.

# Correlation Analysis of Adverse Reactions of Antiosteoporosis Drugs by Different Mechanisms with Bone Turnover and Vitamin D

**DOI:** 10.1155/2021/5402949

**Published:** 2021-10-12

**Authors:** Xiaoling Zhou, Xin Li, Tingting Wei, Ying Xu, Chen Lei

**Affiliations:** ^1^Department of Nephrology, General Hospital of Ningxia Medical University, Yinchuan, Ningxia 750004, China; ^2^Department of Endocrinology, General Hospital of Ningxia Medical University, Yinchuan, Ningxia 750004, China

## Abstract

**Objective:**

The risk factors for the most common adverse reactions of two types of antiosteoporosis drugs in the first treatment of postmenopausal osteoporosis were analyzed to investigate the relationship between the occurrence of adverse reactions and different bone transition states and vitamin D levels.

**Methods:**

A total of 381 postmenopausal women who were diagnosed with osteoporosis in the Osteoporosis Clinic of Ningxia Medical University General Hospital from January 2017 to June 2020 were enrolled. A telephone follow-up survey was conducted on the mentioned subjects. According to the survey results, the mentioned subjects were selected according to their first use of antiosteoporosis drugs. They were divided into zoledronic acid and teriparatide acetate groups. The subjects in the two groups were divided into two groups according to the presence or absence of adverse reactions after medication and according to vitamin D level and P1NP level, and the correlation between the two factors and the occurrence of adverse reactions was analyzed.

**Results:**

Among the 307 patients treated with zoledronic acid for antiosteoporosis, 99 patients developed acute phase adverse reactions (APR+), accounting for 32.2% of the total subjects. 56.7 percent of the subjects had vitamin D deficiency. The 25(OH)D level of the APR + subjects was 16.75 ± 9.20 ng/mL, significantly lower than that of the APR− patients (23.68 ± 10.67 ng/mL). Serological P1NP level in APR+ patients was 73.95 ± 34.50 ng/ml, significantly higher than that of APR− patients with 55.80 ± 36.91 ng/ml. Musculoskeletal symptoms were observed in 14 of the 74 subjects treated with teriparatide acetate, accounting for 18.9% of the total subjects. The 25(OH)D level was deficient in 59.5% of the subjects. The 25(OH)D level of the subjects with musculoskeletal symptoms was 15.96 ± 8.17 ng/ml, while that of the subjects without musculoskeletal symptoms was 20.86 ± 8.52 ng/ml, which showed no statistical significance. The reason was considered to be related to the small sample size included in the study. The P1NP level of subjects with musculoskeletal symptoms was 96.85 ± 58.52 ng/ml, significantly higher than the P1NP level of subjects without musculoskeletal symptoms (55.28 ± 27.87 ng/ml).

**Conclusions:**

The 25(OH)D level in vivo was negatively correlated with the acute phase adverse reactions after the first infusion of zoledronic acid. When the rate of bone formation is increased and osteoblasts are active, the risk of acute phase adverse reactions is increased with the use of zoledronic acid as antiosteoporosis therapy. There was no significant correlation between 25(OH)D levels and musculoskeletal symptoms after teriparatide acetate treatment of osteoporosis. When the rate of bone formation is increased and osteoblasts are active, the risk of adverse reactions to musculoskeletal symptoms is increased with antiosteoporosis treatment with teriparatide acetate.

## 1. Introduction

Osteoporosis (OP) is a systemic bone disease marked by reduced bone strength and increased risk of fracture [1]. Women lose about 30%–40% of their peak bone mass during their lifetime [2]. The diagnosis rate of OP in China is 66.7%, and only less than 25% of people have received effective antiosteoporosis treatment [3].

There are many kinds of antiosteoporosis drugs, and the two types of representative antiosteoporosis drugs with different mechanisms are bone resorption inhibitors and bone formation promoters which are used the most in clinical practice. Studies have shown that, after the first infusion of zoledronic acid, 42.4% of patients experienced acute phase adverse reactions (APR) with mild or moderate severity, which generally occurred within 24–36 h after use and relieved within 72 h [4, 5]. According to the classic ACTive test [6–8], the representative of bone-enhancing drugs is teriparatide acetate, which often has side effects with musculoskeletal symptoms such as limb pain. Therefore, this study aims to analyze the relationship between vitamin D, bone turnover marker P1NP, and adverse reactions of anti-osteoporosis drugs, analyze the risk factors of the most common adverse reactions of two osteoporosis drugs in the treatment of postmenopausal osteoporosis, and study the occurrence of adverse reactions under different bone turnover and the correlation between vitamin D levels.

## 2. Materials and Methods

### 2.1. Study Design and Participants

A total of 381 postmenopausal women, aged 63.83 ± 9.45 years, who were diagnosed with osteoporosis in the Osteoporosis Clinic of Ningxia Medical University General Hospital from January 2017 to June 2020 were enrolled. All the subjects were treated with antiosteoporosis drugs, including 307 patients (age: 63.03 ± 9.34 years) who were first treated with zoledronic acid and 74 patients (age: 67.14 ± 9.21 years) who were treated with teriparatide acetate. Telephone follow-up includes general information (including age, height, weight, etc.) and collection of part of the patient's clinical data (including adverse reactions to antiosteoporosis drug treatment, etc.). In the 307 patients treated for the first time, 99 patients developed acute phase adverse reactions and were assigned to the experimental group, accounting for 32.2% of the total study subjects, while the remaining 208 subjects were assigned to the control group. In the 74 subjects treated with teriparatide acetate, 14 developed musculoskeletal symptoms and were assigned to the experimental group, accounting for 18.9% of the total subjects, while the remaining 60 subjects were assigned to the control group.

Written informed consent was obtained from all patients, with the following exceptions: (1) patients who have been previously treated with bisphosphonates or other drugs that affect bone metabolism; (2) patients with related diseases affecting bone metabolism; (3) patients with bone pain caused by diseases related to the rheumatic immune system; (4) people with recent fever, muscle and joint pain, sore throat, and other related symptoms caused by infectious diseases; (5) patients with some neuromuscular system diseases that affect the results of bone mineral density measurement; (6) severe liver and renal insufficiency; (7) all patients with a history of malignant tumor; (8) having a history of serious smoking and alcohol abuse; and (9) being in a coma or delirious or unable to cooperate.

### 2.2. Methods

According to diagnostic, inclusion, and exclusion criteria, 381 postmenopausal patients (age: 63.83 ± 9.45 years) with osteoporosis were enrolled in the study, which were divided into the zoledronic acid group and the teriparatide acetate group based on the first use of antiosteoporosis drugs.

#### 2.2.1. Zoledronic Acid

Telephone follow-up was used to collect general information of the 307 study subjects and the conditions during the follow-up: The results included age, weight, height, body mass index (kg/m^2^), menopausal years, and the occurrence of acute adverse reactions. VAS pain scoring was used to score the patients and the score was recorded. The outpatient medical records of the research subjects were retrieved through HIS system of our hospital, and other general information and clinical biochemical indicators (including serum calcium, parathyroid hormone, P1NP, 25 hydroxyl vitamin D, *T* value of bone mineral density, etc.) were recorded before the first infusion of zoledronic acid. All the subjects were forbidden from eating food and drinking water after 9 pm on the day before the blood sample collection and kept fasting for 10 hours. Four venous blood samples, each 5–10 ml, were collected at 8 am on the second day and detected by the same chemiluminescence method in the biochemical laboratory of our hospital. P1NP levels were determined by enzyme-linked immunoassay.

All subjects in the zoledronic acid group were given domestic zoledronic acid injection 5 mg intravenously after blood samples were collected, and the infusion time was more than 15 minutes. From the day of infusion to the next 3 days, adverse reactions of the subjects were recorded through telephone follow-up. APR is characterized by a transient mild influenza-like syndrome, such as fever, sore throat, catarrh symptoms, muscle, and arthralgia, which usually develops within 24 to 36 hours after the first infusion and subsides spontaneously within 2 to 3 days. The criteria for inclusion in the experimental group were as follows: (1) fever caused by other infectious factors which was excluded with armpit temperature as the standard and body temperature ≥37.3°C; (2) transient influenza-like symptoms including transient nasal congestion, headache, sore throat, runny nose, and other catarrh symptoms; (3) musculoskeletal symptoms including muscle pain and bone pain intensification. Muscle pain manifested as chest, waist and back, limb muscle, and joint pain. According to the VAS score (visual analog pain score method) to determine the patient's pain level [12], on the ruler of marked VAS score, with the poles with digital “0” and “10,” “0” indicating painless and “10” indicating the highest level of pain, the complaints of the gold standard for research object, according to the complaints of the expression, in the rule table corresponding position, for the pain scores. The higher the value, the higher the pain grade of the patient. The pain from low grade to high grade was aggravated bone pain.

The patients were divided into the acute phase adverse reaction group (APR+ group) and the nonacute phase adverse reaction group (APR− group) according to whether or not they had acute phase adverse reaction. The APR+ group consisted of 99 subjects, accounting for 32.2% of the total subjects, as the experimental group. The other 208 subjects were the control group. The subjects in APR+ group and APR− group were divided into vitamin D deficiency ≤20 ng/ml, vitamin D deficiency of 21–29 ng/ml, and vitamin D deficiency ≥30 ng/ml according to their levels of 25 hydroxyvitamin D (25(OH)D), respectively. The correlation between VD level and APR was analyzed using SPSS 26.0 statistical software. The subjects in APR+ group and APR− group were divided into normal or decreased P1NP group and elevated P1NP group according to the difference of their P1NP serological levels. The correlation between P1NP level and APR was analyzed.

#### 2.2.2. Teriparatide Acetate

Telephone follow-up was conducted to collect general data of 74 subjects and their conditions during follow-up, including age, weight, height, body mass index (kg/m^2^), menopausal years, and musculoskeletal symptoms, and VAS pain scale was used to determine and record the score. Then, the outpatient medical records of the subjects were retrieved through HIS system of our hospital, and other general information and clinical biochemical indicators (including serum calcium ions, 25 hydroxyl vitamin D, parathyroid hormone, P1NP serological level, bone mineral density, *T* value, etc.) were recorded before the injection of teriparatide acetate. All the subjects were forbidden from eating food and drinking water after 9 pm on the day before the blood sample collection and kept fasting for 10 hours. Four venous blood samples, each 5–10 ml, were collected at 8 am on the second day and detected by the same chemiluminescence method in the biochemical laboratory of our hospital. P1NP levels were determined by enzyme-linked immunoassay. All subjects in the teriparatide acetate group were also injected with teriparatide acetate 20μg/time, 1 time/day, subcutaneously after blood collection, the injection site was the abdominal wall or thigh, and the treatment was for at least 1 month. Follow-up by telephone was used to record whether the subjects had musculoskeletal symptoms during use, and the criteria for inclusion in the experimental group included the aggravation of muscle pain and bone pain. Muscle pain manifested as chest, waist and back, limb muscle, and joint pain. According to the VAS score (visual analog pain score method) to determine the patient's pain level [12], on the ruler of marked VAS score, with the poles with digital “0” and “10,” “0” indicating painless and “10” indicating the highest level of pain, the complaints of the gold standard for research object, according to the complaints of the expression, in the rule table corresponding position, for the pain scores. The higher the value, the higher the pain grade of the patient. The pain from low grade to high grade was aggravated bone pain.

According to the presence or failure of musculoskeletal symptoms, the patients were divided into musculoskeletal symptoms+ group and musculoskeletal symptoms− group. A total of 14 subjects in the musculoskeletal symptoms+ group were the experimental group, accounting for 18.9% of the total subjects, and the remaining 60 subjects were the control group. Subjects in the musculoskeletal symptoms+ group and musculoskeletal symptoms− group were divided into vitamin D deficiency ≤20 ng/ml, vitamin D deficiency 21–29 ng/ml, and vitamin D deficiency ≥30 ng/ml according to their levels of 25 hydroxyvitamin D (25(OH)D), respectively. The association between VD levels and musculoskeletal symptoms was analyzed using SPSS 26.0 statistical software in three groups with sufficient vitamin D (≥30 ng/ml). The subjects in the musculoskeletal symptoms+ group and the musculoskeletal symptoms− group were divided into the normal or decreased P1NP group and the elevated P1NP group according to the difference in serum levels of P1NP (amino terminal peptide of type I procollagen). The group criteria were the zoledronic acid group. The relationship between P1NP level and APR was analyzed using SPSS 26.0.

#### 2.2.3. Statistical Analysis

The measurement data was expressed as mean ± standard deviation ($\bar{x}$ ± *s*). SPSS 26.0 statistical software was used to process the data, and descriptive statistical analysis was performed on the baseline measurement values. Analysis of variance (ANOVA) and Wilcoxon rank-sum test of continuous variables were used to compare the demographic characteristics and biochemical parameters of bone turnover between the adverse reactions group and the nonadverse reactions group. The classification variables were analyzed by the chi-square test and Fisher's exact probability method of bidirectional disordered *R∗C* table data. Analysis of covariance (ANCOVA) was used to adjust for the values of any confounding factors. Logistic regression analysis was used to study the relationship between 25(OH)D level and adverse reactions and the relationship between P1NP level and adverse reactions, and the potential confounders were adjusted at *P* < 0.05, where the difference is considered significant.

## 3. Results

### 3.1. Results of the Study on Zoledronic Acid

Of the 307 patients in the zoledronic acid group, 32.2% developed acute phase adverse reactions (APR). There were no significant differences between APR+ and APR− groups in age, height, weight, BMI, Ca, PTH, and BMD *T* values. The two groups were comparable. The level of 25(OH)D in APR+ group was significantly lower than that in APR− group. The level of P1NP in APR+ group was significantly higher than that in APR− group (Table 1).

Among the 99 patients with APR+ in the zoledronic acid group, 76.8% had a deficient 25(OH)D level. The level of 25(OH)D was insufficient in 14.1% of patients. Only 9.1% (9/99) of patients had adequate 25(OH)D levels. Of the 208 subjects with APR−, 47.1% had deficient 25(OH)D levels. The 25(OH)D level was inadequate in 31.7% of the patients. The 25(OH)D level was adequate in 21.2% (44/208) of the patients (Figure 1). Among the 99 patients with APR+ in the zoledronic acid group, 52.5% had normal or decreased serological P1NP levels. Serological P1NP levels were elevated in 47.5% of patients. Serological P1NP levels were normal or decreased in 81.2% of the 208 subjects with APR−. The serum P1NP level was elevated in 18.8% of patients (Figure 2).

The chi-square test was conducted on the stratified classification variables of vitamin D, and the results showed that 25(OH)D levels were divided into three groups: ① VD ≤ 20 ng/ml; (2) 21–29 ng/ml; and (3) ≥30 ng/ml. The comparison of the three groups (*P* < 0.01) showed that the difference was statistically significant, indicating that the incidence of APR was different under different 25(OH)D levels. The results of pairwise comparison of the three groups were as follows: between groups ① and ② and between groups ① and ③, the difference was statistically significant (*P* < 0.01), and the incidence of APR was different. There was no significant difference in >0.05 between groups ② and ③ (Table 2).

Chi-square test was carried out for P1NP classification variables with different levels, and the following conclusions were drawn: ① normal or reduced P1NP group and ② P1NP elevated group. The comparison of groups ① and ② (*P* < 0.01) showed that the difference was statistically significant (Table 3).

Logistic regression was used to analyze the positive and negative correlations between vitamin D level and P1NP risk factors and adverse reactions. The results showed that vitamin D level was negatively correlated with adverse reactions. There was also a positive correlation between P1NP level and adverse reactions (Table 4).

### 3.2. Results of Teriparatide Acetate Group Study

Musculoskeletal symptoms occurred in 18.9% of the 74 subjects in the teriparatide acetate group. There were no significant differences in age, height, weight, BMI, Ca, PTH, and BMD *T* values between the group with musculoskeletal symptoms (musculoskeletal symptoms+ group) and the group without musculoskeletal symptoms (musculoskeletal symptoms− group). The levels of 25(OH)D in the musculoskeletal symptom+ group were lower than those in the musculoskeletal symptom− group. The level of P1NP in the musculoskeletal symptom+ group was significantly higher than that in the musculoskeletal symptom− group (Table 5).

Of the 14 subjects with musculoskeletal symptoms+ in the teriparatide acetate group, 71.4% had deficient 25(OH)D levels. In 21.4% of patients, 25(OH)D levels were inadequate. Only one patient had an adequate 25(OH)D level. Among the 60 patients with nonmusculoskeletal symptoms, 56.7% of the patients had deficient 25(OH)D levels. 25(OH)D levels were inadequate in 28.3% of the patients; 25(OH)D levels were adequate in 15% of patients (Figure 3). Among the 14 subjects with musculoskeletal symptoms in the teriparatide acetate group, 28.6% of the patients had normal or reduced serological P1NP levels. The serum P1NP level was elevated in 71.4% of the patients. Serological P1NP levels were normal or decreased in 70% of the 60 patients with nonmusculoskeletal symptoms. Serological P1NP levels were elevated in 30% of patients (Figure 4).

The classification variables of vitamin D stratification were statistically analyzed by Fisher's exact probability method in *R∗C* table. The results showed that 25(OH)D levels were divided into three groups: ① VD ≤ 20 ng/ml; (2) VD = 21–29 ng/ml; and (3) VD ≥ 30 ng/ml. Groups ①, ②, and ③ showed no significant difference (*P*=0.760 and *P* < 0.05), indicating that there was no difference in the incidence of musculoskeletal symptoms after antiosteoporosis treatment with teriparin at different levels of 25(OH)D. There was no significant difference in the incidence of musculoskeletal symptoms after antiosteoporosis treatment with teriparatide acetate when the serum level of 25(OH)D was ≤20 ng/ml, 21–29 ng/ml, and ≥30 ng/ml (Table 6).

Chi-square test was carried out for P1NP classification variables with different levels, and the following conclusions were drawn: ① normal or reduced P1NP group and ② P1NP elevated group. The comparison of groups ① and ② (*P*=0.04 and *P* < 0.01) showed that the difference was statistically significant (Table 7).

Logistic regression analysis of the positive and negative correlations between vitamin D level and two risk factors of P1NP and adverse reactions showed that there was no correlation between vitamin D level and adverse reactions. There was a positive correlation between P1NP level and adverse reactions (Table 8).

## 4. Discussion

OPF is the most serious consequence of osteoporosis, most commonly occurring in the vertebral body, pelvis, proximal humerus, distal radius, and other parts of the spine, among which vertebral fractures are the most common [10]. Studies have shown [11] that, in 2010, it was estimated that about 2 million cases of osteoporotic fractures occurred in China, costing more than 900 million US dollars, and about 1.85 million cases of female fractures occurred, which are three times those of male fractures, and the cost accounts for 76% of the total fracture cost. Clearly, the treatment of osteoporosis and its complications poses a major challenge to the economic and medical resources of countries and societies.

At present, the conservative treatment of osteoporotic fractures still plays an important role. Most of the patients with pure osteoporotic vertebral compression fractures will choose conservative treatment under the condition that their work and life are not seriously affected. Both zoledronic acid and teriparatide acetate have different pharmacological mechanisms in the treatment of osteoporosis, but there is a risk of some adverse reactions during the treatment process, which affects the patient's dependence and drug efficacy to some extent. Literature has shown that the occurrence rate of APR is between 30% and 50% during the first infusion of zoledronic acid [12]. At present, relevant studies have shown that there is a close relationship between the level of 25(OH)D in vivo and the adverse reactions of zoledronic acid [6]. In this study, the subjects were divided into zoledronic acid group and teriparatide acetate group according to the different anti-OP drugs used. Each group was divided into experimental group and control group according to the presence or absence of adverse reactions. The present study found that VD levels were deficient in 56.7% of 307 patients treated with zoledronic acid. The level of 25(OH)D in the zoledronic acid APR+ group was significantly lower than that in the APR− group, suggesting that, to reduce the incidence of APR after the infusion of zoledronic acid, the serum level of 25(OH)D should be supplemented to 21.70 ng/mL, which is far below the level of vitamin D required to prevent the occurrence of APR. B. Francesco et al. [6] studied the curve representing the relationship between vitamin D levels and fever, and higher vitamin D levels may be required to prevent APR induced by zoledronic acid infusion. Is there any association between vitamin D levels and adverse reactions after teriparatide acetate treatment of osteoporosis? In this study, the results showed that there was no correlation between vitamin D levels and musculoskeletal symptoms after teriparatide acetate treatment of OP. However, due to the small number of people using this drug, it is not sufficient to fully analyze the association between vitamin D and musculoskeletal symptoms. Therefore, a larger sample is needed to verify the correlation between vitamin D and musculoskeletal symptoms after the use of teriparatide acetate.

Bone transition markers (BTMs) identify types of OP, predict rate of bone loss, assess risk of brittle fracture, determine bone transition status, and assess drug response and patient compliance [1]. The study of Xiaofeng Li et al. [9] showed that the choice of drugs for OP patients can be guided by bone transformation markers. In other words, when the level of bone transformation is low, drugs that promote bone formation should be selected. At high bone turnover levels, osteoresorption suppressor drugs should be chosen. This has great clinical implications for drug selection in OP patients. However, at present, in addition to effectiveness, there are some studies on safety, and there are few literatures on the correlation between different bone transition states and adverse reactions of antiosteoporosis drugs. In the present study, 381 patients treated with anti-OP drugs were analyzed and their pretreatment P1NP levels were recorded. It was found that the rate of adverse reactions was higher in both zoledronic acid and teriparatide acetate treated with anti-OP drugs than in a group with normal or reduced bone formation rate. Combined with Xiaofeng Li et al.'s research results, this study, from the perspective of safety, further supports Xiaofeng Li's conclusion; that is, under the condition of high bone turnover, the use of drugs that inhibit bone resorption can rapidly inhibit bone metabolism indexes and reduce the rate of bone turnover. Therefore, the reduction of bone turnover rate can reduce the occurrence of adverse reactions to a certain extent, which is beneficial for osteoporosis patients. Studies have confirmed [13] that when bone formation markers are reduced by half and bone resorption markers are reduced by 70%, the corresponding risk of nonvertebral fracture is reduced by about 44% and 40%, respectively. In this study, only bone formation markers were selected as bone conversion markers, represented by P1NP, but not bone resorption markers, which could not fully reflect the state of bone conversion. Therefore, the experimental results of this study can only indicate that, in the state of active osteogenesis, the incidence of adverse reactions of two types of anti-OP drugs with different mechanisms is clearly higher than that in the normal or reduced bone formation state. In the follow-up safety analysis of antiosteoporosis drugs, we expect to see a comprehensive study on how different bone transition states affect adverse reactions to drugs.

## Figures and Tables

**Figure 1:** Percentage of 25(OH)D deficiency in patients in the zoledronic acid group.

**Figure 2:** Serum P1NP levels of patients in the zoledronic acid group.

**Figure 3:** Percentage of 25(OH)D deficiency in patients in the teriparatide acetate group.

**Figure 4:** Serum P1NP levels of patients in the teriparatide acetate group.

**Table 1:** Baseline demographics and characteristics (*n*, $\bar{x}$ ± *s*).

Factors	All patients	APR−	APR+	*p*
Age (years)	63.03 ± 9.34	62.8 ± 8.96	63.52 ± 10.13	0.634
Height (cm)	160.16 ± 6.28	160.28 ± 6.70	159.92 ± 5.30	0.436
Weight (kg)	62.47 ± 5.04	62.13 ± 4.80	63.18 ± 5.48	0.088
BMI (kg/m^2^)	24.41 ± 2.21	24.25 ± 2.21	24.73 ± 2.19	0.076
Ca (mmol/l)	2.38 ± 0.09	2.38 ± 0.09	2.37 ± 0.10	0.244
PTH (pg/ml)	42.34 ± 15.46	41.11 ± 14.74	44.92 ± 16.67	0.065
25(OH)D (ng/ml)	21.45 ± 10.71	23.68 ± 10.67	16.75 ± 9.20	<0.01
P1NP (ng/ml)	61.65 ± 37.08	55.80 ± 36.91	73.95 ± 34.50	<0.01
*T* value	−2.7 ± 0.1	−2.71 ± 0.09	−2.7 ± 0.11	0.092

*Note.* APR+ : acute adverse reactions; APR−: no acute adverse reactions; P1NP: amino terminal peptide of type I procollagen; *T* value: bone mineral density *T* value.

**Table 2:** Comparison of different vitamin D levels in the zoledronic acid group (*n*, %).

VD (ng/ml)	APR+ (*n*)	APR− (*n*)	*c* ^2^	*P*
≤20 ng/ml	76	98	24.023	<0.01
21–29 ng/ml	14	66		
≥30 ng/ml	9	44		

**Table 3:** Comparison of zoledronic acid groups according to different P1NP levels (*n*, %).

P1NP (ng/ml)	APR+ (*n*)	APR− (*n*)	*c* ^2^	*P*
P1NP normal or decreased group	52	169	27.445	<0.01
P1NP elevated group	47	39		

**Table 4:** Logistic regression analysis of VD, P1NP, and adverse reactions in zoledronic acid group (*n*, %).

Risk factor	Regression coefficient	Standard error	OR	*P*
Vit. D	−0.76	0.017	0.927	<0.01
P1NP	0.011	0.004	1.011	0.005

**Table 5:** Baseline demographics and characteristics (*n*, $\bar{x}$ ± *s*).

Factors	All patients	Musculoskeletal symptoms+	Musculoskeletal symptoms−	*P*
Age (years)	67.14 ± 9.21	68.71 ± 10.92	66.77 ± 8.83	0.48
Height (cm)	158.30 ± 3.01	159.29 ± 2.85	158.08 ± 3.03	0.218
Weight (kg)	61.97 ± 3.96	60.79 ± 4.48	62.25 ± 3.81	0.215
BMI (kg/m^2^)	24.75 ± 1.73	23.96 ± 1.81	24.93 ± 1.67	0.059
Ca (mmol/l)	2.39 ± 0.10	2.43 ± 0.16	2.39 ± 0.08	0.173
PTH (pg/ml)	41.26 ± 15.01	39.26 ± 16.27	41.72 ± 14.81	0.553
25(OH)D (ng/ml)	19.93 ± 8.62	15.96 ± 8.17	20.86 ± 8.52	0.052
P1NP (ng/ml)	63.14 ± 38.81	96.85 ± 58.52	55.28 ± 27.87	0.003
*T* value	−2.7 ± 0.10	−2.7 ± 0.12	−2.7 ± 0.09	0.499

**Table 6:** Comparison of teriparatide acetate group with different vitamin D levels (*n*, %).

VD (ng/ml)	Musculoskeletal symptoms+ (*n*)	Musculoskeletal symptoms− (*n*)	*c* ^2^	*P*
≤20 ng/ml	10	34	0.856^a^	0.76
21–29 ng/ml	3	17		
≥30 ng/ml	1	9		

*Note.* ^a^The value of Fisher's exact test (*R* × *C*).

**Table 7:** Comparison of teriparatide acetate groups according to different P1NP levels (*n*, %).

P1NP (ng/ml)	Musculoskeletal symptoms+ (*n*)	Musculoskeletal symptoms− (*n*)	*c* ^2^	*P*
P1NP normal or decreased group	4	42	8.283	0.004
P1NP elevated group	10	18		

**Table 8:** Logistic regression analysis of VD, P1NP, and adverse reactions in teriparatide acetate group.

Risk factors	Regression coefficient	Standard error	OR	*P*
Vit. D	−0.075	0.052	0.928	0.144
P1NP	0.028	0.011	1.028	0.011

## Data Availability

The data can be obtained from the corresponding author upon reasonable request.
